# Self-Medication Practices, Prevalence, and Associated Factors among Syrian Adult Patients: A Cross-Sectional Study

**DOI:** 10.1155/2022/9274610

**Published:** 2022-06-28

**Authors:** Rawan N. K. Abdelwahed, Manaf Jassem, Ayham Alyousbashi

**Affiliations:** ^1^Dermatology and Venereology University Hospital, Ministry of Higher Education, Damascus, Syria; ^2^Department of Internal Medicine, Damascus Hospital, Ministry of Health, Damascus, Syria; ^3^Department of Pediatrics, Damascus Hospital, Ministry of Health, Damascus, Syria

## Abstract

**Objectives:**

Self-medication (SM) means using drugs to treat self-diagnosed diseases or symptoms. Despite its important role in reducing the load on medical services, it may bear many risks. This study aims to determine the prevalence of SM and its determinants among adult inpatients of Damascus Hospital, Syria. *Study design.* Cross-sectional study.

**Methods:**

453 adult inpatients were asked to complete a questionnaire through face-to-face interviews. Data were analysed using statistical package for the social sciences (SPSS). A chi-square test was used to detect correlation between variables.

**Results:**

Out of 453 respondents, 67.3% practiced self-medication. Most used drugs were analgesics, antipyretics, and antibiotics. The main indications for SM included headache, cough/flu, and body aches. Pharmacists were the main source of knowledge about the drugs used in SM. The leading reason for practicing SM was the mildness of the complaint. Approximately half of the participants declared they read leaflets of drugs they used in SM. In this study, SM was significantly associated with monthly income, age, and living place.

**Conclusions:**

The prevalence of SM in Damascus Hospital is high. Larger, nationwide studies are needed to identify the prevalence and determining factors of SM in Syria and to suggest the appropriate measures to control this phenomenon.

## 1. Introduction

The World Health Organization (WHO) defines self-medication as the use of drugs to treat self-diagnosed disorders or symptoms, or the intermittent or continued use of a prescribed drug for chronic or recurrent diseases or symptoms [1]. Self-medication may involve using over-the-counter (OTC) medications, prescription-only medicines, or complementary and alternative medicines [2].

Despite its important role in care of minor illnesses [3, 4], and its ability to reduce the load on medical services and constrain treatment costs, SM cannot be considered a completely safe practice [1], and it may give rise to many medical problems such as antibiotic resistance, misdiagnosis, use of excessive drug dosage, prolonged duration of use, drug interactions, and polypharmacy [5].

Recent studies conducted in different parts of the world such as Egypt [3], Jordan [4], Lebanon [6], Palestine [7], Vietnam [8], and Brazil [9], vary in their estimation of the percentage of patients who practice self-medication, with prevalence rates that range from about 16.1% to 83.3%. Studies indicate that the use of self-medication is influenced by several factors, such as sociodemographic factors, level of education, and the availability of pharmacies [10].

In Syria, self-medication, as a research topic, has not received the attention it deserves; a literature review yielded one study conducted in Syria on the prevalence of self-medication among undergraduate medical students in two universities [11]. To our best knowledge, no studies on the prevalence of self-medication among hospital patients have been conducted.

Data on the prevalence of, and factors associated with, self-medication in Syria are necessary to plan interventions aimed at improving the self-use of medicines in the country and limiting the risks associated with practicing self-medication.

This study aims to determine the prevalence of self-medication among adult patients attending Damascus Hospital, Syria; to identify factors that could influence the practice of self-medication; to identify classes of medications used; to identify sources of information regarding medications used; and to recognize reasons for self-medication.

## 2. Methods

### 2.1. Study Design

This is a cross-sectional, survey-based study that was conducted between August and September 2020 among adult patients of Damascus Hospital, the main hospital affiliated with the Ministry of Health, located in Damascus, the capital of Syria.

### 2.2. Sample Size and Sampling Technique

The sample size (*n*) was determined using the equation of one proportion: [*n* = *Z*2 P (1-P)/d2], with the following assumptions: *Z* = 1.96 for 95% confidence level, prevalence of self-medication (P) = 0.62 (62%), margin of error (d) = 0.05. P value was determined after conducting a pilot study on 50 patients at Damascus Hospital. Applying the previous formula resulted in a sample size (*n*) of 362. In order to have more accurate results, we decided to set the sample size (*n*) to 453 patients. To collect the required surveys, systematic random sampling was used. First, we contacted the admission office of Damascus Hospital to get a list of all the patients admitted between August and September 2020; the total number of patients admitted during this period (N) was 1359 patients. After that, we calculated the sampling interval (*k*) using the formula: [*k* = *N*/*n*]. Applying the formula resulted in a sampling interval (*k*) of 3. We chose the starting point to be the 2^nd^ patient in the list of admitted patients and selected every 3^rd^ patient till we got the desired sample size.

### 2.3. Ethical Approval and Consent to Participate

The study was approved by the scientific and ethical committee of Damascus Hospital, and all necessary permissions were obtained prior to starting the study. The patients were informed on the aim and objectives of the study and written informed consents were obtained from them prior to data collection. Participants were also informed that participation in the study is voluntary, and the data was assured to be anonymous and confidential.

### 2.4. Instruments and Data Collection

An English questionnaire was constructed following a literature review [12–14]. It was then revised by public health and research experts to ensure its relevance to the study. Because Arabic is the native language in Syria, the questionnaire was translated to Arabic by an expert translator, translated back to English, and validated for consistency.

Data was collected through face-to-face interviews by 8 trained data collectors. Surveys were completed after clarifying the purpose of the study to the participants and obtaining written informed consent from them.

The questionnaire included two sections: (1) demographic characteristics of patients; 2. practicing self-medication, types of drugs used, treated symptoms, source of information about self-medication, reasons for self-medication, self-medication outcome, knowledge of side effects of self-medication drugs, and attitudes towards self-medication.

### 2.5. Statistical Analysis

Data were analysed using SPSS software version 22. Descriptive statistics were applied to represent the demographics of the sample and to describe self-medication behaviors using counts, percentages, and means. The chi-square test was used to detect association between sociodemographic data and self-medication practice, the outcome of self-medication, and drugs used. A *P* value of  < 0.05 was considered statistically significant.

## 3. Results

### 3.1. Sociodemographic Characteristics

453 participants completed the questionnaire; the majority of them were 41–60 years old (47.4%). 180 participants (39.7%) were males and 273 (60.3%) were females. Most of the participants lived in the countryside (65.9%), within 30–60 minutes from the hospital (46.5%), earned less than 48 US dollars per month (48.1%), received primary education (48.3%), and were nonsmokers (56.8%). Sociodemographic characteristics of the participants are shown in Table 1.

### 3.2. Self-Medication Prevalence and Practices

Of the sample studied, 304 subjects (67.3%) practiced self-medication in the three months preceding the study, with most of them practicing self-medication more than five times (66.1%). 182 individuals (57.2%) were not aware of the side effects of the drugs they used to self-medicate. More than half of the participants (54%) declared that they had read the associated pamphlets. The majority (91%) noted that self-medication helped them alleviate their symptoms or cure their illness. When asked about what they would do if self-medication failed, 146 individuals (54.9%) said they would seek medical consultation for further investigation and management of their complaint. Regarding individuals' opinion on the safety of practicing self-medication, 321 (70.9%) said they consider it not safe, and 237 (52.3%) said they would not recommend other people to self-medicate (Table 2).

### 3.3. Self-Medication Drugs, Indications, and Information Sources

The drug groups most commonly used for self-medication among participants were analgesics (55.7%), antipyretics (15.3%), and antibiotics (11.1%) (Table 3).

Predominant indications for self-medication included headaches (28.7%), cough/flu (16%), and body aches (14%) (Table 4).

The majority of participants received information about drugs they used to self-medicate from pharmacists (35.2%), while 22.8% had previous knowledge or experience of their ailment.

Most of the participants practiced self-medication because they considered their complaint mild and did not indicate medical consultation (22.7%); other notable reasons included economic reasons (20.4%), and previous experience with the complaint (15.9%).

### 3.4. Factors Associated with Self-Medication

Self-medication was significantly associated with monthly income (*P* = 0.021), age (*P* = 0.004), and living area (*P* = 0.026); patients younger than 40 years old, those who lived in the city, and those who earned more than 48 US dollars per month were more likely to self-medicate. Although the prevalence of self-medication among females was higher compared to males (70.32% versus 62.2%), no significant association was found between practicing self-medication and gender (*P* = 0.066). In addition to that, no association was found between practicing self-medication and participants' level of education (*P* = 0.214), though most of the participants who practiced self-medication did not reach high school level. Furthermore, no association was found between practicing self-medication and smoking (*P* = 0.613), nor employment status (*P* = 0.619) (Table 5).

## 4. Discussion

This study indicates that practicing self-medication (SM) is common in Damascus Hospital, with a prevalence of 67.3% in the preceding three-month period. While this prevalence rate is higher than that in Jordan (42.5%) [4], Brazil (16.1%) [9] and Ethiopia (50.2%) [15], it is notably lower than that of Lebanon (79.1%) [6], Palestine (87%) [7], Egypt (73%) [3], Vietnam (83.3%) [8], and Pakistan (84.4%) [16]. This variation might be explained by different recall periods, healthcare services, the economic situation, and social and cultural factors.

Association between sociodemographic factors and self-medication was minor in this study. Practicing self-medication was slightly higher among females than males. Although a strong association was found between gender and SM in many studies, no significant association was found in this study. This also remains a worldwide point of debate because females were more involved in self-medication practice in some societies [6, 9, 17], while males were predominant in others [8, 18].

Self-medication practice was more prominent in ages younger than 40 years old, and a strong association was found between age and SM. This contradicts with a study conducted in Egypt in which self-medication was prevalent in ages older than 40 years old [3], while it associates with other studies held in Saudi Arabia [17], Lebanon [6], and Brazil [9] which also revealed a predominance in younger ages.

In this study, higher monthly income was related to the practice of self-medication, unlike the results of studies conducted in Ethiopia [15] and China [19] which showed an association with lower income. Moreover, residents of the city were more likely to practice self-medication than those of the countryside, which relates to a study conducted in Erbil [20]. This might be justified by the abundance of pharmacies in cities compared to the countryside, which facilitates access to drugs.

Analgesics, antipyretics, and antibiotics were the most common drug classes used in self-medication. This resembles the findings of a Lebanese study, in which acetaminophen-based analgesics (48.7%), nonsteroidal anti-inflammatory drugs (24.6%), and antibiotics (8.8%) were the most commonly used drugs in self-medication [6], but differs from the results of another study conducted in Syria which indicated that the use of antitussives and vitamins was more common than antibiotics [11]. These dissimilarities might be justified by the difference between populations studies, as the latter only targeted undergraduate medical students, so their medical knowledge might have played a role in their using less antibiotics. This high prevalence of antibiotics use should be repressed as antibiotic resistance is jeopardizing public health in Syria [21] and the government should fight the unprescribed use of antibiotics.

Headaches, cough/flu, and body aches were the main conditions to treat. These findings came in concordance with those of a study in Saudi Arabia [17] in which headaches, flu, and cough were the predominant indications. However, fever was also a predominant indicatior in Saudi Arabia, while suffering from body aches was more common in our study.

The leading reasons for self-medication were the mildness of the illness and the elevated cost of medical consultations, followed by having previous knowledge or experience of the illness. Similar reasons were evident in other studies [3, 6, 7]. The increased fear of high treatment costs could be justified by the deterioration of economic status in Syria in the light of the current war [22].

Pharmacists were the main source of advice on which drugs to use in self-medication. Their role as an alternative to medical consultation was also prominent in other studies [3, 6, 15]. This might be explained by the expensiveness of healthcare services, prolonged waiting periods in clinics and hospitals, and the abundance of, and ease of access to, pharmacies.

More than half of the respondents stated that they read the associated medication pamphlets, which are mandatory for all medicines in Syria, compared with only one-third in an Eritrean study [15]. Furthermore, half of the participants lacked knowledge about the side effects of commonly used medications. This was also noted in a study held in Lebanon where 64.5% of the participants lacked this knowledge [6]. This difference between the percentage of people who read pamphlets and those who knew the side effects of commonly used drugs might be justified by the low educational level of many of the participants, which limits their ability to understand medical language used in pamphlets. Encouraging physicians and pharmacists to explain the probable side effects of medications may be warranted in such cases.

The majority declared that self-medication helped them alleviate their symptoms. The effectiveness of self-medication was also noted in a study held in China with 94.5% of the participants noticing an improvement [19]. This might encourage the action of practicing self-medication as beneficial outcomes are frequently gained. In the case of self-medication failure, more than half of the participants indicated that they would visit healthcare facilities for medical consultation. This good attitude was more prevalent than other actions such as double dosing or repeating the same medication and was correlated with the results of other studies [15].

Fortunately, about two thirds declared that self-medication is not safe and more than half would not recommend it to other people to self-medicate. This contradicts an Indian study in which the majority of people who self-medicated considered self-medication harmless and would advise others to self-medicate [18].

### 4.1. Limitations of This Study

This is a single-center study conducted on a limited number of hospital patients. However, it is worth noting that it is one of the largest hospitals in Damascus, the capital of Syria, and it receives patients from all over the country. Furthermore, this is a cross-sectional study, so it does not address the difference in self-medication patterns among different seasons.

Using surveys depends on self-reported data and is subject to individuals' responses. Also, the nature of face-to-face interviews might have made the participants reluctant to admit wrong attitudes, but emphasizing on the confidentiality of participants' identities and data might have limited this effect. Moreover, the study has focused on the three-month period preceding the interview, which may increase the effect of recall bias.

Surprisingly, the participants in the study were mostly of low education level. Therefore, the results of this study may not reflect the attitudes and practices of people with higher education, and further studies are needed to investigate their practices.

## 5. Conclusion

This study has highlighted the high prevalence of self-medication in Damascus Hospital. The most commonly used drugs were analgesics, antipyretics, and antibiotics. The main conditions to treat were headaches, cough/flu, and body aches. The most common reason for self-medication was the mildness of the ailment. Pharmacists were the main source of information about self-medication.

Because of the limited size of the sample and the fact that this is a single-center study, further nationwide studies are needed to assess the prevalence of the self-medication phenomenon and suggest solutions and measures to control it and limit its undesirable effects.

This study did not address self-medication in special cases like pregnancy, parental medication, and higher education populations.

## Figures and Tables

**Table 1:** Sociodemographic characteristics of participants.

Characteristic	*n* (%)
Age (In years)	
18–25	22 (4.9)
26–40	160 (35.8)
41–60	212 (47.4)
61–85	53 (11.9)

Gender	
Male	180 (39.7)
Female	273 (60.3)

Living area	
City	154 (34.1)
Countryside	298 (65.9)

Smoking	
No	256 (56.8)
Yes	195 (43.2)

Distance from hospital (In minutes)	
Less than 30 minutes	78 (17.3)
30–60 minutes	210 (46.5)
More than 60 minutes	164 (36.3)

Educational Level	
Illiterate	66 (14.6)
Able to read and write	34 (7.5)
Primary school	219 (48.3)
High school	56 (12.4)
Intermediate or higher institute certificate	28 (6.2)
University degree	47 (10.4)
Master or PhD	3 (0.7)

Marital status	
Single	82 (18.3)
Married	384 (77.7)
Divorced	8 (1.8)
Widowed	10 (2.2)

**Table 2:** Other characteristics of self-medication.

Characteristic	*n* (%)
Practicing self-medication in the preceding three months	
No	148 (32.7)
Yes	304 (67.3)

Frequency of self-medication in the preceding three months	
One time	42 (13.0)
Two to five times	67 (20.8)
More than five times	213 (66.1)

Reading associated pamphlets	
No	148 (46.0)
Yes	174 (54.0)

Outcome of self-medication	
Healing of disease	49 (17.0)
Alleviation of symptoms	213 (74.0)
No benefit	26 (9.0)

Actions taken when self-medication fails	
Seeking medical consultation	146 (54.9)
Double dosing	33 (12.4)
Repeating the same drug	33 (12.4)
Waiting for symptoms to resolve on its own	28 (10.5)
Using a stronger drug	15 (5.6)
Using traditional medicine	11 (4.1)

Do you think self-medication is safe?	
Strongly agree	20 (4.4)
Agree	75 (16.6)
Neutral	37 (8.2)
Disagree	210 (46.4)
Strongly disagree	111 (24.5)

Would you recommend others to self-medicate?	
No	237 (52.3)
Yes	216 (47.7)

**Table 3:** Types of drugs used for self-medication.

Drug type	*n* (%)
Analgesics	280 (55.7)
Antipyretics	77 (15.3)
Antibiotics	56 (11.1)
Antihistamines	13 (2.6)
Antacids	12 (2.4)
Cough medicines	7 (1.4)
Flu medicines	9 (1.8)
Antispasmodics	9 (1.8)
Laxatives	3 (0.6)
Antidiarrheals	2 (0.4)
Antiemetics	1 (0.2)
Others (oral contraceptives, ocular and nasal drops, local skin medicines, and herbal medicines)	34 (6.8)

**Table 4:** Indications for self-medication.

Complaint	*n* (%)
Headache	226 (28.7)
Cough and flu	126 (16)
Fever	61 (7.8)
Body aches	110 (14)
Digestive complaints	62 (7.9)
Toothache	57 (7.2)
Allergy	25 (3.2)
Skin infections	20 (2.5)
Dysmenorrhea	11 (1.4)
Other	39 (4.9)

**Table 5:** Association between sociodemographic variables and practicing self-medication.

Variable	Yes, for self-medication	Percentage (CI 95%)	*P* value^*∗*^
Gender			
Male	112	36.8	0.066
Female	192	63.2	

Monthly income (In US dollars)			
Less than 48 US dollars	134	44.1	0.021
More than 48 US dollars	170	55.9	

Educational Level			
Lower than high school	243	91.7	0.214
Higher than high school	22	8.3	

Smoking			
No	175	57.8	0.613
Yes	128	42.2	

Age (In years)			
Less than 40 years	135	45.3	0.004
More than 40 years	163	54.7	

Employment status			
Unemployed	146	48.2	0.619
Employed	157	51.8	

Living area			
City	114	37.6	0.026
Countryside	189	62.4	

Distance from hospital (In minutes)			
Less than 30 minutes	58	19.1	0.247
30–60 minutes	138	46.6	
More than 60 minutes	107	36.4	

^*∗*^ *P*value < 0.05 is considered significant.

## Data Availability

Datasets used/generated during this study are available on reasonable request.
